# Tongyang Huoxue Decoction (TYHX) Ameliorating Hypoxia/Reoxygenation-Induced Disequilibrium of Calcium Homeostasis and Redox Imbalance via Regulating Mitochondrial Quality Control in Sinoatrial Node Cells

**DOI:** 10.1155/2021/3154501

**Published:** 2021-08-10

**Authors:** Xing Chang, Shunyu Yao, Qiaomin Wu, Yanli Wang, Jinfeng Liu, Ruxiu Liu

**Affiliations:** Guang'anmen Hospital, China Academy of Chinese Medical Sciences, Beijing 100053, China

## Abstract

Sick sinus syndrome (SSS) is a disease with bradycardia or arrhythmia. The pathological mechanism of SSS is mainly due to the abnormal conduction function of the sinoatrial node (SAN) caused by interstitial lesions or fibrosis of the SAN or surrounding tissues, SAN pacing dysfunction, and SAN impulse conduction accompanied by SAN fibrosis. Tongyang Huoxue Decoction (TYHX) is widely used in SSS treatment and amelioration of SAN fibrosis. It has a variety of active ingredients to regulate the redox balance and mitochondrial quality control. This study mainly discusses the mechanism of TYHX in ameliorating calcium homeostasis disorder and redox imbalance of sinoatrial node cells (SANCs) and clarifies the protective mechanism of TYHX on the activity of SANCs. The activity of SANCs was determined by CCK-8 and the TUNEL method. The levels of apoptosis, ROS, and calcium release were analyzed by flow cytometry and immunofluorescence. The mRNA and protein levels of calcium channel regulatory molecules and mitochondrial quality control-related molecules were detected by real-time quantitative PCR and Western Blot. The level of calcium release was detected by laser confocal. It was found that after H/R treatment, the viability of SANCs decreased significantly, the levels of apoptosis and ROS increased, and the cells showed calcium overload, redox imbalance, and mitochondrial dysfunction. After treatment with TYHX, the cell survival level was improved, calcium overload and oxidative stress were inhibited, and mitochondrial energy metabolism and mitochondrial function were restored. However, after the SANCs were treated with siRNA (si-*β*-tubulin), the regulation of TYHX on calcium homeostasis and redox balance was counteracted. These results suggest that *β*-tubulin interacts with the regulation of mitochondrial function and calcium release. TYHX may regulate mitochondrial quality control, maintain calcium homeostasis and redox balance, and protect SANCs through *β*-tubulin. The regulation mechanism of TYHX on mitochondrial quality control may also become a new target for SSS treatment.

## 1. Introduction

Sick sinus syndrome (SSS), also known as sinoatrial node dysfunction, is a syndrome of arrhythmias caused by the pathological changes of sinoatrial node (SAN) and its adjacent tissues. It is one of the most refractory major cardiovascular diseases in clinic [1]. With population aging, the incidence of SSS is increasing. SAN, the physiological pacemaker of the heart, can trigger and regulate the rhythm of the heart [2, 3]. Cardiac rhythm is produced by the special cardiac myocytes of SAN and transmitted to the whole atrium and ventricle through the cardiac conduction system. Studies have found that calcium homeostasis and oxidative stress can affect SAN function directly [4]. Mitochondrial quality control (MQC) is closely related to calcium homeostasis and redox balance [5, 6], which directly affect the survival level of sinoatrial node cells (SANCs). Mitochondrion, as the central organelle of apoptosis pathway, is also the main site of tricarboxylic acid cycle and oxidative phosphorylation [7]. Its normal structure and function can meet the energy requirements of heart beating and ejection function, maintaining the homeostasis of intracellular environment, and regulating cell growth [8, 9].

Mitochondria can maintain the normal electrophysiological and contractile functions of cardiomyocytes and SANCs by producing adenosine triphosphate (ATP) and directly participate in the regulation of calcium homeostasis in SANCs. As the main site of ROS production and the first target of ROS attack, excessive ROS production can lead to dysfunction of mitochondrial respiratory electron-transport chain and further affect the balance of redox in cells [10]. Therefore, under the stimulation of hypoxia, inflammation, and high glucose, it will lead to excessive production of ROS and induce structural and functional abnormalities of mitochondria, including imbalance of mitochondrial energy metabolism, reduction of mitochondrial biosynthesis, and abnormal opening of mitochondrial membrane permeability transition pore (mPTP) [11, 12].

Moreover, the dysfunction of the balance system of intracellular “calcium release” and “calcium contraction” can also lead to abnormal increase of intracellular calcium concentration or calcium overload, which can cause the disorder of mitochondrial oxidative phosphorylation [13, 14]. Moreover, high concentration of Ca^2+^ in cytoplasm can increase Ca^2+^ uptake by mitochondria, which will lead to calcium phosphate deposition in mitochondria, and then affect ATP synthesis [15]. Calcium overload can further activate calcium-dependent proteases, promote the transformation of xanthine dehydrogenase into xanthine oxidase, and increase the production of ROS [16, 17]. Therefore, the redox imbalance and mitochondrial dysfunction caused by calcium overload will form a vicious circle and further participate in the process of cell damage [18, 19]. Early correction of mitochondrial dysfunction and regulation of calcium homeostasis and redox balance are important targets for protecting SANCs.

Tongyang Huoxue Decoction (TYHX) has been used in clinic for more than 50 years. It is composed of *Astragalus membranaceus*, ginseng, *Rehmannia glutinosa*, *Angelica sinensis*, and licorice. Many studies have reported that ginsenoside Rb1, resveratrol and astragaloside IV in *Astragalus membranaceus*, ginseng, *Rehmannia glutinosa*, and *Angelica sinensis* can protect mitochondria and regulate redox balance and mitochondrial quality control [20, 21]. Our previous experimental study also found that astragaloside IV, an active ingredient of TYHX, can shorten the action potential duration of injured SANCs in rabbits and protect the cytoskeleton [22]. However, the specific mechanism of TYHX in protecting SANCs and regulating the electrophysiological function of SANCs has not been elucidated. Therefore, this study is aimed at exploring the protective pharmacological action of TYHX on SANCs.

## 2. Materials and Methods

### 2.1. Drugs and Concentration Selection

All Chinese herbal medicines are provided by the pharmacy department of Guang'anmen Hospital. TYHX is composed of five herbs: *Astragalus membranaceus*, ginseng, *Rehmannia glutinosa*, *Angelica sinensis*, and licorice. Decoct all the herbs for 45 minutes, then filter out the solution, then add 6 times the volume of water to decoct again for 30 minutes, and then filter again. Finally, mix the two portions of filtered solution in a 75°C water bath. Finally, 1 g/ml TYHX stock solution was obtained. Correct the pH value to 7.4~7.6, and after centrifugation in a centrifuge, autoclave the supernatant at 8 pounds of pressure for 15 minutes, and then filter with a filter and microporous membrane before use. The nontoxic concentration of the drug was detected by the MTT method, and it was found that 50 *μ*g/ml was the optimal nontoxic concentration of TYHX.

### 2.2. Reagents

DMEM was purchased from GIBCO (USA); FBS and trypsin were purchased from GIBCO (USA); collagenase II, Triton X-100, and Na2EDTA were purchased from Sigma Aldrich; preparation of anoxic hypoxia medium (in mM) is as follows: put 1.8 CaCl_2_, 20 HEPES, 10 KCl, 1.2 MgSO_4_, 98.5 NaCl, 6 NaHCO_3_, 0.9 NaH_2_PO_4_, and 40 sodium lactate in an anoxic chamber at 37°C for 3 h to induce hypoxia; preparation of reoxygenation medium (in mM) is as follows: 1.8 CaCl_2_, 5.5 glucose, 20 HEPES, 5 KCl, 1.2 MgSO_4_, 129.5 NaCl, 20 NaHCO_3_, and 0.9 NaH_2_PO_4_ at 37°C, and finally expose it to an atmosphere with 95% O_2_ and 5% CO_2_ for 2 h.

### 2.3. Isolation of SANCs

A total of 80 rabbits were selected (born time < 24 hours). The rabbits were sterilized with 75% ethanol before operation, and the suckling rabbits were anesthetized with isoflurane. The heart was completely exposed under the anatomical microscope. The SAN tissue was collected from the venous sinus and anterior vena cava root in the middle of the end ridge (2 mm × 2 mm × 2 mm). The tissue was placed in DMEM. The SAN tissue was washed with PBS and cut into pieces (0.3 mm × 0.3 mm × 0.3 mm). Discard the supernatant, add 0.08% trypsin (8 ml) to the chopped tissue for digestion, and shake in 37°C water bath for 5 minutes. After precipitation, the supernatant was removed and discarded, and the tissue was further digested with 8 ml 0.025% collagenase II. The supernatant was collected after sedimentation and transferred to a 50 ml centrifuge tube (containing 20 ml DMEM which contains 15% FBS), following the same procedure three times. The supernatant after digestion was collected and filtered by metal sieve (400 meshes). The supernatant after filtrate centrifuged for 7 min at 940 R/min. The supernatant was discarded after centrifugation, leaving cells suspended in the medium with a density of 1 × 10^5^, which were seeded in 5 culture dishes. The culture dishes were incubated in the cell incubator for 90 minutes. After removing fibroblasts by the differential adhesion method, the remaining cells continued to grow after adding 5-bromo-2′-deoxyuridine (5-BrdU). After culturing for 24 hours, replace the medium, and then replace it every other day. When replacing the medium, add 5-BrdU (0.1 mmol L^−1^) [22].

### 2.4. Grouping and Culturing of Cells

Before the experiment, SANCs were divided into 5 groups: (1) control group: cells were cultured under the above normal conditions; (2) H/R group: cells were cultured in hypoxic medium instead of DMEM (as shown in the section on reagents) and placed in a hypoxic environment for 3 hours. Replace the hypoxic medium with the reoxygenated culture medium (as shown in the section on reagents), and place it in an environment with 95% O_2_ and 5% CO_2_ to continue the culturing; (3) TYHX group: SANCs were pretreated with TYHX before H/R modeling; (4) TYHX + siRNA-*β*-tubulin group: SANCs were treated with *β*-tubulin siRNA (siRNA-*β*-tubulin) before modeling and drug treatment; and (5) TYHX + Ad-*β*-tubulin group: SANCs were treated with an adenoviral vector (Ad-*β*-tubulin) overexpressing *β*-tubulin before modeling and drug treatment.

### 2.5. Apoptosis Detection

The SANCs in each group were washed with PBS. Then, an apoptosis detection kit was used for detection. Flow cytometry and the CXP software (Beckman, Brea, CA, USA) were used for analysis.

### 2.6. ROS

SANCs were incubated with 2′,7′-dichlorofluorescein (10 *μ*m) at 37°C for 20 min. Then, the fluorescence was measured by a fluorescence microscope (Olympus, Japan) and a flow cytometry (Beckman, Brea, CA, USA). The ROS in the cells was detected by flow cytometry.

### 2.7. Determination of Antioxidant Enzyme Activity and MDA Level

The SOD\MDA\GSH-Px\TrxR kit was provided by Nanjing Jiancheng Institute of Biological Engineering. All operations were carried out in accordance with the manufacturer's instructions. Simply put, cells were collected before and after modeling and drug pretreatment. After ultrasonic treatment, the cell lysate was centrifuged at 3000°C 20 r/min, and then the supernatant was collected to determine the level of SOD\MDA\GSH-Px\TrxR.

### 2.8. Cellular Energy Metabolism

The oxygen consumption rate (OCR) of the whole cell was analyzed by an XFp extracellular flux analyzer (Seahorse Biosciences) to detect the basic respiration, respiratory reserve, maximum respiration, ATP production level, and proton leakage level of mitochondria. SANCs (5 × 10^5^ cells/well) were inoculated. Mitochondrial respiration was detected, and mitochondrial energy metabolism was recorded according to the manufacturer's instructions.

### 2.9. Laser Confocal and Immunofluorescence

After simulated H/R, cells were rinsed with PBS, then fixed with 4% paraformaldehyde. The treated cells were placed in a 37°C wet box, into which 100 *μ*l of the first antibody was added, and the cells were incubated at 4°C for 16 hours. The cells were rinsed with PBS for four times, each time for 5 minutes. Then, the second antibody was added, and the cells were incubated in the dark for 1 hour. After buffering glycerin was added, the fluorescence image and fluorescence intensity were detected and analyzed by a laser confocal microscope. The average fluorescence intensity was analyzed by the ImageJ software.

### 2.10. Calcium Release/Calcium Contraction Detection

After SANCs were collected in an EP tube, 0.1% BSA low-calcium solution containing Fluo-4 AM was used to prepare the incubation solution and then cultured at 37°C for 20-30 min. Then, the solution was centrifugated to remove the fluo-4 AM working fluid. A small amount of SANCs were placed in a confocal dish coated with laminin. The concentration of Ca^2+^ was recorded.

### 2.11. Real-Time PCR

TRIzol was used to extract the total RNA of each group. Under the catalysis of reverse transcriptase, the total RNA in each group was used as template to synthesize cDNA by reverse transcription. The PrimeScript™ RT Kit was used to reverse transcribe RNA into cDNA with a gDNA eraser. Real-time quantitative PCR was used with cDNA as template, and the data was analyzed by 2^−ΔΔCT^.

### 2.12. Western Blot

Western Blot was used to study the protein expression of SERCA2a/RyR2/CaV1.3/NCX/*β*-tubulin (*β*-tubulin, Abcam, ab6046; SERCA2a, Abcam, ab150435; RyR2, Abcam, ab21796; Cav1.3, Abcam, ab84811; and NXC, Abcam, ab177952). The total protein was obtained from the SANCs. Protein samples are separated on 8% and 12% SDS-PAGE gel and transferred to nitrocellulose membranes. Transfer the protein to the PVDF membrane, block it with 5% skimmed milk powder at room temperature for 1 hour, and then incubate it with the primary antibody overnight at 4°C. The cells were incubated with the first antibody overnight. The ImageJ software was used to analyze the data by optical density analysis.

### 2.13. Statistical Analysis

The data obtained by the SPSS 22.0 statistical software were applied, and normal distribution data were measured by the *X* ± *S*-form expression. Median or quartile was used for nonnormal distribution data, and *t*-test was used for paired or two groups of continuous measurement data. One-way analysis of variance is used to compare multiple sets of data, and two groups with SNK-q. The nonparametric test was used for nonnormal data, and *χ*^2^ test was used for pairwise comparison of classification data. The significance standard was *p* < 0.05.

## 3. Results

### 3.1. TYHX Can Effectively Improve the Activity of SANCs and Inhibit Apoptosis

We first verified the effect of TYHX on activity of SANCs, and it was found that TYHX can further improve cell viability through CCK-8 detection (Figure 1(a)), while effectively inhibiting cell apoptosis (Figures 1(e) and 1(f)). In order to further verify the role of skeleton protein (*β*-tubulin) in SANC damage induced by hypoxia/reoxygenation (H/R), we detected the levels of *β*-tubulin by PCR/Western Blot and immunofluorescence. It was found that H/R can reduce the mRNA and protein expression levels of SANCs, and TYHX can reverse this phenomenon (Figures 1(b) and 1(c)), so it was inferred that the mechanism of TYHX to improve the viability of SANCs may be related to *β*-tubulin. To further verify this hypothesis, SANCs were treated with an adenoviral vector overexpressing *β*-tubulin (Ad-*β*-tubulin) and *β*-tubulin siRNA (siRNA-*β*-tubulin). Then, through CCK-8 and cell apoptosis detection, it was found that SANCs treated with siRNA-*β*-tubulin eliminated the protective effect of TYHX on SANCs (Figures 1(d)–1(f)). However, the SANCs treated with Ad-*β*-tubulin under the intervention of TYHX further increased the protective effect of TYHX on SANCs (Figures 1(d)–1(f)). The experimental results suggest that TYHX can protect against H/R-induced SANC damage. The protective effect of TYHX on SANCs may be accomplished through the regulation of *β*-tubulin, and the specific mechanism needs further verification.

### 3.2. TYHX Inhibits H/R-Induced Overproduction of ROS in SANCs and Regulates the Redox Balance

SAN is the normal pacing point of the heart, and its lesion was directly shown by abnormal pacing function or aggravated SAN fibrosis. Although the SANCs themselves consume little oxygen, the loss of redox balance caused by the extremely low oxygen concentration may be the main cause of SANC damage. In order to further clarify the protective mechanism of TYHX on H/R-induced SANCs damage, we tested the level of ROS production in SANCs and the activity of oxidative stress marker MDA through ROS production level detection and ELISA. We also tested the activity of antioxidant enzyme superoxide dismutase (SOD), glutathione peroxidase (GSH-Px), and thioredoxin reductase (TrxR). The study found that compared with the control group, SANCs treated with H/R significantly enhanced ROS production and the activity of MDA, while the activity of SOD, GSH-Px, and TrxR was significantly weakened (Figures 2(a)–2(h)). TYHX can inhibit ROS production and the activity of MDA and enhance the activity of SOD, GSH-Px, and TrxR (Figures 2(a)–2(h)). However, ROS production and MDA activity of SANCs treated with siRNA-*β*-tubulin were significantly enhanced, while the activity of SOD, GSH-Px, and TrxR was significantly weakened (Figures 2(a)–2(h)). Ad-*β*-tubulin can improve the regulation of TYHX on redox balance (Figures 2(a)–2(h)). The above results indicate that TYHX can inhibit the level of ROS production, regulate the activity of MDA/SOD/GSH-Px/TrxR, and maintain the internal redox balance of SANCs. The mechanism by which TYHX maintains the redox balance may be closely related to the regulation of *β*-tubulin.

### 3.3. TYHX Regulates H/R-Induced Calcium Homeostasis Disorder in SANCs through SERCA2a/RyR2/CaV1.3/NCX

Oxidative stress can lead to abnormal energy metabolism and directly affect calcium influx or calcium release from endoplasmic reticulum through the opening of calcium ion channel. Therefore, in order to further verify that the protective mechanism of TYHX on SANCs is related to its regulation of calcium homeostasis disorder in SANCs, we detected the calcium release level of SANCs by laser Flow cytometry and confocal scanning. The results showed that the calcium release level of SANCs was significantly increased after H/R treatment. However, TYHX pretreatment could significantly inhibit calcium release (Figures 3(a) and 3(b)). It is worth noting that calcium release in the siRNA-*β*-tubulin + TYHX group was significantly higher than that in the TYHX group. And in ad-*β*-tubulin + TYHX group, the calcium release of SANCs was significantly decreased (Figures 3(a) and 3(b)). The results showed that TYHX could inhibit the H/R-induced calcium overload and maintain calcium homeostasis in SANCs.

SERCA2a and RyR2 play a crucial role in the regulation of intracellular calcium homeostasis, and CaV1.3/NCX can also regulate the role of calcium channel to maintain the normal level of calcium release. In order to further verify the mechanism of TYHX-regulating calcium homeostasis, we further verified the mRNA and protein expression levels of SERCA2a/RyR2/CaV1.3/NCX by PCR and Western Blot. The experimental results showed that compared with the normal group, the mRNA and protein expression levels of RyR2 in SANCs treated with H/R were significantly increased, while the mRNA and protein expression levels of SERCA2a, CaV1.3, and NCX were significantly reduced (Figures 3(c) and 3(d)). TYHX can reverse this phenomenon, increase the mRNA and protein expression levels of SERCA2a/CaV1.3/NCX, and inhibit the mRNA and protein expression level of RyR2 (Figures 3(c) and 3(d)). However, the mRNA and protein expression levels of SERCA2a, CaV1.3, NCX, and RyR2 in the siRNA-*β*-tubulin + TYHX group were significantly lower than those in the TYHX group, while those in the Ad-*β*-tubulin + TYHX group were on the contrary (Figures 3(c) and 3(d)). The above results indicate that TYHX can maintain intracellular calcium homeostasis of SANCs by regulating the balance of SERCA2a and RyR2 and that of CaV1.3/NCX, and its regulation mechanism may be directly related to the regulation of backbone protein (*β*-tubulin).

### 3.4. TYHX Ameliorates H/R-Induced SANC Damage by Regulating Mitochondrial Energy Metabolism

As a key part of ROS attack and imbalance of calcium homeostasis, mitochondria play an important role in the protective mechanism of H/R-induced SANC damage. We tested the function of mitochondrial respiratory chain (mainly mitochondrial respiratory complex I/III) and the level of mitochondrial energy metabolism through ELISA and the hippocampal detection system. At the same time, we also tested the opening rate of mitochondrial membrane permeability transition pore (mPTP). Studies have found that H/R can inhibit the expression level of SANC mitochondrial respiratory complex I/III (Figures 4(a) and 4(b)), while further inhibiting mitochondrial basal respiration, maximum respiration, respiratory reserve, and ATP synthesis, increasing the level of proton leakage and the opening level of mPTP (Figures 4(c)–4(h)). TYHX can reverse these phenomena, improve mitochondrial energy metabolism and mitochondrial respiratory chain function, and inhibit the abnormal opening of mPTP (Figures 4(c)–4(h)). It is worth noting that the treatment of SANCs with siRNA-*β*-tubulin and Ad-*β*-tubulin + TYHX can directly affect the regulation of TYHX on the mitochondrial energy metabolism, as well as the function of mPTP (Figures 4(a)–4(h)). In order to further explore the effect of mitochondrial capacity metabolism on calcium homeostasis of SNC, we detected the expression level of NCX1.1 by immunofluorescence and found that the expression level of NCX1.1 in H/R group was decreased, and the intervention of TYHX could increase the expression level of NCX1.1, siRNA-*β*-tubulin, and Ad-*β*-tubulin + TYHX which can directly affect the regulation of TYHX on the calcium homeostasis (Figure 4(i)). The above results indicate that TYHX can increase the level of mitochondrial energy metabolism, regulate the function of mitochondrial respiratory chain, and protect SANCs, but its regulation of mitochondrial quality control needs further verification.

### 3.5. TYHX Ameliorates H/R-Induced SANC Damage by Regulating Mitochondrial Quality Control

Mitochondrial quality control includes mitochondrial biosynthesis, fusion and fission, and mitochondrial autophagy which removes damaged and aged mitochondria and synthesizes new mitochondria. MQC can maintain mitochondrial renewal and protect mitochondrial function. In order to verify that TYHX can regulate mitochondrial quality control in SANCs, we detected Fis1, Mfn1, Tfam, and PGC1*α* by PCR. The mRNA levels of the two groups were compared. ATG5 and Parkin were also detected. It was found that the expression level of Fis1 was increased and that of Mfn1, Tfam, and PGC1*α* was decreased in H/R group (Figures 5(a)–5(d)). The mRNA expression levels of ATG5 and Parkin were inhibited (Figures 5(e) and 5(f)). In the TYHX group, the expression of Fis1 was inhibited while that of Mfn1, Tfam, and PGC1*α* was increased (Figures 5(a)–5(d)). The mRNA expression level of ATG5 and Parkin was further increased (Figures 5(e) and 5(f)). The results indicate that H/R can lead to mitochondrial fission/fusion imbalance, enhancing mitochondrial fission while weakening mitochondrial fusion. Both mitophagy and biosynthesis were attenuated. This may be due to the failure to remove or degrade the damaged mitochondria normally due to the rise of mitochondrial fission level. However, TYHX can protect mitochondrial function, regulate mitochondrial dynamics, and improve the efficiency of mitophagy and mitochondrial biosynthesis. Furthermore, mitochondrial membrane potential and TUNEL staining were found that H/R-induced mitochondrial quality control disorder may indirectly lead to the loss of mitochondrial membrane potential (MMP) and cell death (Figures 5(g)–5(k)), while TYHX can restore MMP and maintenance of cell survival (Figures 5(g)–5(k)).

We also found that the mRNA expression level related to mitochondrial quality control was increased or decreased in varying degrees in the siRNA-*β*-tubulin + TYHX group and ad-*β*-tubulin + TYHX group (Figures 5(a)–5(f)). Interestingly, si/ad-*β*-tubulin can also indirectly affect the regulatory effect of TYHX on MMP and cell survival level (Figures 5(g)–5(k)). The results suggest that *β*-tubulin has a certain relationship with the structure or function of mitochondria.

### 3.6. HPLC Analysis of Active Components of TYHX

In order to further verify the active components of TYHX, the main components of TYHX were analyzed by HPLC. Five compounds were identified by different extraction methods: ferulic acid, ginsenoside Rb1, astragaloside IV, diosgenin, and catalpol (Figure 6). Studies have reported that the above five active ingredients from TYHX can play a good therapeutic effect in different types of cardiovascular diseases [20, 23]. Moreover, it can protect many kinds of cells (including endothelial cells, cardiomyocytes, and sinoatrial node cells) under stress conditions [20]. The protective mechanism may be closely related to the mitochondria quality control. As shown in Figure 7, a variety of active ingredients in TYHX can regulate Parkin/ATG-led mitophagy. Inhibit the expression of Fis1, increase the expression of Mfn on the mitochondrial membrane, and promote the occurrence of mitochondrial fusion. And by adjusting PGC1*α* and Tfam to improve the mitochondrial biosynthesis effect, adjust the mitochondrial quality control and the calcium homeostasis mechanism dominated by SERCA2a and RyR2, restoration of sinoatrial node cell activity.

## 4. Discussion

In this study, we found that TYHX can significantly improve mitochondrial energy metabolism, regulate the function of mitochondrial respiratory chain, inhibit the abnormal opening of mPTP and the excessive production of ROS, and improve the activity of antioxidant enzymes. For the regulation of calcium homeostasis, TYHX can increase the mRNA and protein expression levels of SERCA2a, CaV1.3, and NCX, inhibit the mRNA and protein expression levels of RyR2, and maintain the expression level of *β*-tubulin. It can inhibit the calcium overload and apoptosis of SANCs and improve the activity of SANCs. After treating with siRNA-*β*-tubulin, the protective effect of TYHX on SANCs and the regulation of mitochondrial quality control were eliminated, and calcium overload and oxidative stress were aggravated. After treating with ad-*β*-tubulin, the protective effect of TYHX on SANCs was further strengthened. Therefore, we infer that *β*-tubulin is an important way for TYHX to improve the activity of SANCs.

“Calcium Clock” is the process by which the sarcoplasmic reticulum automatically releases Ca^2+^ to control automatic depolarization [24]. The core of the “Calcium Clock” lies in the balance of the sarcoplasmic reticulum RyR2 and SERCA2a on the release and uptake of Ca^2+^. The “Calcium Clock” plays an important role in the physiological mechanism of SANC pacing [25]. When the “Calcium Clock” depolarizes, it induces the opening of L-type Ca^2+^ channels. The ryanodine receptors (RyR2) that triggers SR release a large amount of Ca^2+^, causing membrane ion current and calcium-activated current activity, and at the same time, generating action potentials, guiding SANCs to pace, and conducting the heart's beating function [26, 27]. Once the physiological process of “calcium release” and “calcium contraction” loosed balance, it will lead to calcium homeostasis disorder, which makes SANC pulsation dysfunction or induces excessive proliferation of fibroblasts and induces SAN fibrosis [28, 29]. This experimental study has confirmed that TYHX can regulate and maintain the balance of SERCA2a and RyR2, increase the mRNA and expression of the calcium-regulating molecule CaV1.3/NCX, and maintain calcium homeostasis.

Ca^2+^ transport proteins include endoplasmic reticulum calcium release proteins, mitochondrial outer membrane, and mitochondrial inner membrane-related proteins [30]. Mitochondria can take up calcium ions released from the endoplasmic reticulum via mitochondria-associated endoplasmic reticulum (MAM). The release of calcium ions from the endoplasmic reticulum is mainly mediated by RyRs (ryanodine receptors) [31, 32]. Then, the mitochondria calcium uniporter (MCU) mediates calcium ions to cross the outer mitochondrial membrane and the inner mitochondrial membrane and enters the mitochondrial matrix. SERCA is a calcium pump that transports intracellular calcium to the endoplasmic reticulum [33]. The activity and expression of SERCA are essential for maintaining a baseline calcium release or resting intracellular calcium. Various studies have reported the cardioprotective effects of SERCA [12, 34, 35]. The decreased expression of SERCA can mediate endothelial cell necrosis in ischemia-reperfusion. The concomitant malfunction of MCU and mitochondrial membrane permeability transition pore (mPTP) may be an important reason for promoting calcium overload [12]. Under the induction of H/R, the dysregulation of the mitochondrial respiratory chain caused by the imbalance of redox balance and the abnormal opening of mPTP may be the main reasons for the disorder of the regulation mechanism of calcium homeostasis of SERCA and RyRs.

*β*-Tubulin, the most important tubulin in SANCs, functions to maintain the distribution of cytoskeleton, microtubules, cell function, and cell dynamics [36]. *β*-Tubulin also functions to regulate the bioelectric activity of SANCs and maintain the contraction and relaxation of SANCs [37]. The study also found that *β*-tubulin can regulate mitochondrial oxidative phosphorylation and energy flux in the regulation of apoptosis. *β*-Tubulin is directly related to mitochondrial function and is coexpressed with mitochondrial creatine kinase (MtCK) [38]. Moreover, the normal morphological arrangement of mitochondria is also maintained by the cytoskeleton structure, so *β*-tubulin directly affects the integrity of the mitochondrial structure and the normal function of the mitochondria [39]. Studies have also shown that microtubule stabilizers can act on L-type calcium channels through *β*-tubulin to keep the channels open for a long time and extend the open time. After treating the cells with microtubule depolymerization agents, it is found that ICa-L was significantly inhibited. *β*-Tubulin can regulate the expression levels of RyR2 and SERCA2a by regulating ICa-L, participating in the regulation of the “Calcium Clock,” thereby maintaining the electrophysiological balance of SANCs, and the normal physiological functions of SANCs [38]. Our study is consistent with the above results.

As the cell's energy factory, mitochondria provide cells with energy and substrates required for biosynthesis and determine the cell's fate [40]. Abnormal cell metabolism often induces mitochondrial damage, which in turn triggers cell apoptosis through a series of protein signals [41]. Mitochondrial quality control (MQC) is the adaptive regulation of mitochondrial protein turnover and mitochondrial fusion, fission, and mitophagy [42]. The main purpose of MQC is to quickly remove defective mitochondrial fragments and replenish mitochondria in time. These processes can maintain the structure and morphology of mitochondria under stress conditions, thereby maintaining the normal biological functions of cells [43]. Under hypoxic stress, mitochondrial respiratory function and energy metabolism suffer severe imbalance, which is also accompanied by mitochondrial respiratory chain dysfunction. By detecting the gene transcription related to mitochondrial biogenesis and mitochondrial fission/fusion, it is found that under hypoxia, the mitochondria fission/fusion of SANCs loosed balance, suppressing mitophagy and biosynthesis. Therefore, it is inferred that the mitochondrial homeostasis disorder caused by hypoxia will directly affect the MQC and further severely damage the normal structure and function of the mitochondria, but lead to the overproduction of ROS. Excessive production of ROS will further affect the redox balance, resulting to enhanced activity of MDA, a marker of oxidative stress, and weakened activity of SOD, GSH-Px, and TrxR. The further aggravation of cellular oxidative stress and the disorder of calcium homeostasis will lead to a further increase in the apoptosis level of SANCs, which may be the main mechanism of SAN dysfunction.

In addition, the mitochondrial respiratory chain is the main source of mitochondrial ROS. Active oxygen is a by-product of electrons transferred in the respiratory chain. They are mainly NADH-produced: ubiquinone oxidoreductase and cytochrome C (cytC) oxidoreductase in the respiratory chain. The reactive production of excessive ROS can directly damage the mitochondrial respiratory chain function, reduce mitochondrial energy metabolism, destroy the mitochondrial antioxidant system, and further aggravate oxidative stress damage [17]. At the same time, it also induces the increase of mitochondrial calcium release level, the imbalance of calcium homeostasis, and the abnormal opening of the mitochondrial membrane permeability transition pore (mPTP) [44]. The imbalance of ion concentration inside and outside the mitochondria, which may be H/R-mediated mitochondria imbalance in quality control, can indirectly lead to the imbalance of calcium homeostasis. As shown in Figure 7, TYHX can restore mitochondrial respiratory chain function and mitochondrial energy metabolism level, maintain mitochondrial function, adjust the balance of mitochondrial fission/fusion, and ameliorate mitophagy and mitochondrial biosynthesis.

A study in *Nature* also found that NCLX, the mitochondrial sodium-calcium exchanger, or mitochondrial Na^+^/Ca^2+^ exchanger, can affect the function of the heart [45]. Animals lacking NCLX will die, and only 13% of the animals can survive for two weeks. The study confirmed that calcium homeostasis disorder in mitochondria can seriously affect heart function. Inhibiting the uptake of calcium ions can lead to the loss of cardiac stress response. Under stress, the mitochondria of the heart need to take up calcium ions to strengthen cardiac motility. However, excessive uptake of calcium ions can also induce cardiac cell death [45]. This suggests that there may be a basic mechanism for the autonomous balance of “calcium release” and “calcium uptake” in cells or mitochondria. Elrod and his colleagues inhibit the closure of mPTP through genetic manipulation so as to ameliorate the symptoms of sudden death in NCLX knockout mice and maintain the balance mechanism of mitochondrial calcium ion exchange in the heart. They also found that myocardial fibrosis can be limited by reducing the production of ROS [45]. This is consistent with our results. After hypoxia intervention, the calcium release in SANCs increased significantly. This further verified that the balance mechanism of calcium ion exchange in SANCs is closely related to the survival status of cells. TYHX can inhibit the expression of RyR2 by increasing the expression of SERCA2a, NCX, and CaV1.3, thus maintaining the calcium homeostasis in SANCs and protecting SANCs.

Liquid chromatography-mass spectrometry was adopted in the study. TYHX contains ferulic acid, ginsenoside Rb1, astragaloside IV, diosgenin, catalpol, and other active ingredients [46, 47]. Many studies have reported that these drugs have the pharmacological effects of antioxidative stress and regulating MQC. In the process of high-lipid, high-glucose, or anoxia-induced redox imbalance or mitochondrial dysfunction, it can have a good protective effect on cells [48]. Our previous study found that astragaloside IV can increase the expression of HCN4 in injured SANCs of newborn rabbits, protect the damaged cytoskeleton, and improve the survival level of SANCs [22]. Therefore, we infer that the protective effect of TYHX on SANCs may be related to the regulation of the above active ingredients on MQC.

In this study, we have elucidated that the mechanism of TYHX protecting SANCs is closely related to the regulation of calcium homeostasis and MQC, which is of significance to guide the amelioration of sinus syndrome and SAN fibrosis. But at present, this study also has some limitations. Firstly, in the pharmacodynamic study of TYHX, in addition to ferulic acid, ginsenoside Rb1, astragaloside IV, diosgenin, catalpol, and other active ingredients, are there any other active ingredients? This needs further pharmacological research to verify. Secondly, is the regulation of calcium homeostasis and mitochondrial homeostasis by TYHX closely related to drug concentration and dose? Although the concentration gradient screening by CCK-8 was carried out in our experimental study, the effective dose of TYHX needs to be further verified in in vivo study. Finally, TYHX can protect SANCs by regulating mitochondrial homeostasis and calcium homeostasis. As shown in Figure 7, is this closely related to the theory of “balance of yin and yang” in traditional Chinese medicine? This is also the direction of this study and our future research.

## Figures and Tables

**Figure 1:** TYHX can effectively improve the activity of SANCs and inhibit apoptosis of SANCs by preserving *β*-tubulin homeostasis. (a) Cell viability detection (3 group). (b) Laser confocal detection. (c) PCR/Western Blot to detect the level of *β*-tubulin. (d) Cell viability detection (5 group). (e, f) Cell apoptosis level detection, ^∗^*p* < 0.05.

**Figure 2:** TYHX protects SNCs against cellular apoptosis by suppressing oxidative stress and ROS overproduction. (a, b) ROS production detected by flow cytometry. (c) Activity of MDA. (d) Activity of SOD. (e) Activity of GSH-Px. (f) Activity of TrxR. (g, h) ROS production detected by immunofluorescence, ^∗^*p* < 0.05.

**Figure 3:** TYHX regulates H/R-induced calcium homeostasis disorder in SANCs through SERCA2a/RyR2/CaV1.3/NCX. (a) Flow cytometry to detect intracellular calcium release level of SANCs. (b) Laser confocal to detect calcium release from SANCs. (C) PCR to detect the mRNA expression level of SERCA2a/RyR2/CaV1.3/NCX. (D) WB to detect the protein expression level of SERCA2a/RyR2/CaV1.3/NCX, ^∗^*p* < 0.05.

**Figure 4:** TYHX ameliorates H/R-induced SANC damage by regulating mitochondrial energy metabolism/mitochondrial membrane permeability transition pore (mPTP) opening and NCX1.1. (a, b) ELISA to detect the activity of mitochondrial respiratory chain supercomplex I/III. (c–g) ELISA to detect the level of mitochondrial energy metabolism. (h) Open rate of mitochondrial membrane permeability transition pore (mPTP). (i) Immunofluorescence of NCX, ^∗^*p* < 0.05.

**Figure 5:** TYHX ameliorates H/R-induced SANC damage by regulating mitochondrial quality control. (a) mRNA of Fis1 detected by quantitative PCR. (b) mRNA of Mfn1. (c) mRNA of Tfam. (d) mRNA of PGC1*α*. (e) mRNA of Parkin. (f) mRNA of ATG5. (g–i) Mitochondrial membrane potential. (j, k) TUNEL assay for cell death. ^∗^*p* < 0.05.

**Figure 6:** HPLC analysis of active components of TYHX, including ferulic acid, ginsenoside Rb1, astragaloside IV, diosgenin, and catalpol.

**Figure 7:** The mechanism of TYHX-regulating cardiac pacing function through mitochondrial quality control and calcium homeostasis. Figure legend: mitochondrial quality control can regulate the energy metabolism of cells (including endothelial cells, cardiomyocytes, and sinoatrial node cells), mitochondrial oxidative stress signaling pathways, ROS production, redox balance, cell death/apoptosis, calcium homeostasis, and inflammation. An important biological process of the cell growth cycle. H/R can cause phosphorylated Drp1 to accumulate around the outer mitochondrial membrane and induce Fis1-regulated mitochondrial fission. The transient decrease of mitochondrial membrane potential level is accompanied by phosphorylation or dephosphorylation of FUNDC1. The interaction of Parkin and LC3 induces the occurrence of mitophagy. This process is often accompanied by the occurrence of mitochondrial biosynthesis. H/R-induced mitochondrial quality control disorder will further break the balance of mitochondrial calcium release/calcium contraction (regulated by SERCA2a and RyR2), which led to the imbalance of mitochondrial homeostasis and calcium homeostasis. The process of sinoatrial node cell death/apoptosis will be accelerated. A variety of active ingredients in TYHX that can regulate Parkin/ATG-led mitophagy and remove excess mitochondrial fragment. Inhibit the expression of Fis1, increase the expression of Mfn on the mitochondrial membrane, and promote the occurrence of mitochondrial fusion. And by adjusting PGC1*α* and Tfam to improve the mitochondrial biosynthesis effect, adjust the mitochondrial quality control and the calcium homeostasis mechanism dominated by SERCA2a and RyR2.

## Data Availability

The data used to support the findings of this study are available from the corresponding author upon request.
